# MiRNA-574-3p inhibits cell progression by directly targeting CCND2 in colorectal cancer

**DOI:** 10.1042/BSR20190976

**Published:** 2019-12-13

**Authors:** Wen-Cui Li, Yan-Qiong Wu, Bo Gao, Chao-Yun Wang, Juan-Juan Zhang

**Affiliations:** 1 Department of Laboratory Medicine, Taihe Hospital, Hubei University of Medicine, Shiyan 442000, Hubei Province, China; 2 Department of Anesthesiology, Taihe Hospital, Hubei University of Medicine, Shiyan 442000, Hubei Province, China; 3 Reproductive Medicine Center, Taihe Hospital, Hubei University of Medicine, Shiyan 442000, Hubei Province, China

**Keywords:** apoptosis, colorectal cancer (CRC), Cyclin D2 (CCND2), microRNA-574-3p, migration, proliferation

## Abstract

Colorectal cancer (CRC) remains the candidate for one of the typical types of malignant tumors of in gastrointestinal tract all around the world, which leads to tremendous death and ranks as the top leading death of cancer. Recently, microRNAs have emerged as double-edged sword in numerous cancers. This investigation aims to discuss the regulative role of microRNA-574-3p (miR-574-3p), elucidating its molecular mechanism and clinical significance in CRC. Herein, it revealed to us that miR-574-3p was lowly expressed in CRC tissues in comparison with the matched paracarcinoma tissues. In addition, transfection of SW480 and HT29 cells with miR-574-3p mimics prohibited the post-transcriptional expression of Cyclin D2 (CCND2), which then significantly blocked cell growth and cell migration, yet triggered cell apoptosis. Also, dual-luciferase reporter assays proved the role of CCND2 as the targeted gene for miR-574-3p. miR-574-3p overexpression prohibited the activity of CCND2 in SW480 and HT29 cells. Silencing of CCND2 in SW480 and HT29 CRC cell lines leading to reduced cell proliferative and migrative rates, and enhanced apoptotic rate. The suppressive effects of elevation of miR-574-3p on the proliferation of the human CRC cells and promotive effects on cell apoptosis by targeting CCND2 were further illustrated in the *in vitro* studies. Thus, we hypothesize that miR-574-3p may be served as a prospective therapeutic candidate for CRC.

## Introduction

In the present stage, colorectal cancer (CRC) ranks at the top of malignant caners, which leading to about 700,000 deaths per year [1]. Most CRC patients are diagnosed in advanced stages, often results in poor prognosis [2]. More than 10% percent of CRCs were diagnosed in the relatively late stages, such as metastatic stages (stage IV), which lead to low survival rate. However, only a few established diagnostic methods and CRC prognostic biomarkers were available during the last decade. Therefore, it is urgent to uncover new biomarkers to elevate the level of CRC treatment and prognosis and promotes the beneficial effects to patients, especially for those at the stage with high death risk.

MicroRNAs (miRNAs) turn to a group of endogenous regulatory RNAs without coding ability and they are typically with 18–25 nucleotides in length, which modulate the gene expression widely via directly docking to the 3′-UTR of the mRNAs [3]. Approximately, 30–50% of protein-coding genes for humans are deemed to be controlled by miRNAs [4]. miRNAs have been extensively studied to contribute to the onset and development of numerous tumors [5]. Furthermore, miRNAs play important roles in diverse tumor carcinogenic and suppressive processes, including radiotherapy or chemotherapy resistance, tumor viability, metastasis as well as cell cycle [3]. Meanwhile, the relative expression levels of different miRNA in plasma, serum and tumor samples have widely been utilized to accurately identify the types of human cancers, potentiating that miRNA could be a biomarker for the diagnosis of human cancers, as well as for the development of prognosis for patients with cancer [6]. It was indicated that miR-574-3p regulates the cell growth in osteosarcoma and gastric cancer [7,8]. However, it’s still not clear whether miR-574-3p is involved in the progress of CRC. Taken together, the present study focused on the effect of miR-574-3p in CRC cells, which would extensively offer new theoretical knowledge for the therapeutic potential of miRNA in regulating CRC.

## Materials and methods

### Tissue collection

Clinical specimens of cancerous tissues and adjacent tissues from 62 patients with CRC undergoing surgery were collected from Jan 2014 to Oct 2015 at Taihe Hospital, Hubei University of Medicine. Patients recruited in this investigation had accepted no chemotherapy, radiotherapy, immunotherapy or systemic therapy before surgery. The clinical stages of CRC patients were classified by following the criteria established by the Union for International Cancer Control (UICC). All carcinoma samples and paracarcinoma tissues were examined and confirmed by two trained pathologists (Table 1). The recruited patients in the whole studies have signed informed consent documents. The investigation protocol was authorized by the Research Ethics Committee of the Taihe Hospital, Hubei University of Medicine.

**Table 1:** Correlation of miR-574-3p expression with clinicopathological feature of patients with CRC

Parameters	*n*	miR-574-3p expression				*P*
		High	Percentage	Low	Percentage	
Age						
<65	32	15	46.88	17	53.12	0.6402
≥65	30	18	62.00	12	38.00	
Sex						
Male	32	18	56.25	14	43.75	0.5036
Female	30	13	43.33	17	56.67	
Tumor size						
>5 cm	38	13	34.21	25	65.79	0.0080
≤5 cm	24	21	87.50	3	0.125	
Clinical stage						
I/II	40	29	72.50	11	27.50	0.0003
III/IV	22	5	22.73	17	77.27	
Distant metastasis						
Absent	37	13	35.14	24	64.86	0.0148
Present	25	18	72.00	7	28.00	

### Cell lines and culture conditions

Human CRC cell lines SW480, HT29, LOVO and normal intestinal epithelial cells NCM460 were acquired from the commercial products of ATCC (Manassas, VA, U.S.A.) and cultured in DMEM (ATCC) supplemented with 2.5 mm l-glutamine (Sigma, St. Louis, MO, U.S.A.) and 10% FBS (Hyclone, Logan, UT, U.S.A.). All medium contained 100 IU/ml penicillin and streptomycin. All cells were cultured in a constantly humid incubator at 37°C with CO_2_ of 5%.

### qRT-PCR

Total RNA was isolated from tumor tissues by the Trizol reagent (Invitrogen Inc., Carlsbad, CA, U.S.A.) by following the manual offered by the manufacturer. The expression level of miRNA-584-3p was detected with SYBR PrimeScript RNA RT-PCR kit (TAKARA, Dalian, China), which was compared with U6 snRNA expression level. The cDNA was synthesized by reverse transcribed of total RNA (2 μg) with M-MLV reverse transcriptase and then was used for qRT-PCR analysis (Promega, Fitchburg, WI, U.S.A.). In details, QRT-PCR was conducted with SYBR green PCR Master Mix (TOYOBO, Osaka, Japan) on ABI PRISM 7500 sequence detection system. GAPDH was utilized as the reference gene for calculating the relative expression level of mRNA of CCND2 gene. Primers of miRNA and internal control were designed as following: miR-574-3p, F: 5′-ATCGGAAGTTGAGTGAGCCGCGTC-3′, R: 5′-GCCGTGAGTCAGGAGTGGT-3′; CCND2, F: 5′-CATCCTCACGGCCTCGGCT-3′, R: 5′-CGGCGTGTGTTTATCGGAATCCA-3′; GAPDH, F: 5′-CACCTGCGCTGTGTGGACT-3′, 5′-GGATGGCTGATGTGTCGGGTGG-3′. The 2−ΔΔ*C*t method is used to calculate the results and perform analysis.

### Western blot analysis

First, proteins are split on the SDS-PAGE gels and then wet-transferred onto PVDF membranes by electrophoresis (Millipore, Billericay, Massachusetts). Next, Primary antibodies were used to incubate the membranes at 4°C overnight. On the second day, the membranes were washed thoroughly and incubated with the secondary antibody at room temperature for 1 h. The primary antibodies contain cleaved CCND2 (1:1000, Abcam, Cambridge, MA, U.S.A.) and anti-GAPDH (1:1500, Abcam). The secondary antibodies were rabbit-anti-mouse IgG (1:2000, Santa Cruz Biotechnology, Santa Cruz, CA, U.S.A.). ECL Chemiluminescent Detection System (Thermo Fisher Science, Rochester, New York) of the density of each individual protein bands were calculated by using Bio-Rad Quantity One software (Bio-Rad, Hercules, CA, U.S.A.). All triplicate experiments have been done for each of the experiments.

### Plasmid construction

The full length of 3′-UTR of CCND2 gene was clonally inserted into psi-CHECK2 vector (Promega), which was used as 3′-UTR-WT of CCND2 gene. The 3′-UTR mutant of CCND2 was constructed by QuikChange site-directed mutagenesis kit (Stratagene, San Diego, CA, U.S.A.). All plasmids have been confirmed with DNA sequencing.

### Cell transfection

The miR-574-3p simulated sequences and disrupted sequences (NCs) were purchased from Ribobio, Guangzhou, China. siRNA for CCND2 gene (5′-UCAUGAAGAACUUCUGUUGGTT-3′) and the corresponding control gene (5′-UGUAAGUACCCGAGUUUGTT-3′) were bought from Shanghai GenePharma Company. CRC cells (1 × 10^5^) were seeded onto 24-well plates and incubated in the constant incubator for 24 h, which were then transfected into CRC cells with the miR-574-3p mimics (50 mm) or CCND2-siRNA (100 mm). Lipofectamine 2000 (Invitrogen) in the medium shortage of fetal bovine serum (FBS) was used as the transfection reagent in this experiment.

### Luciferase assay

Cells (100 μl) were cultured on 24-well plates, followed by the co-transfection by 100 ng CCND2 3′-UTR-WT co-transfected or mutant psi-CHECK2 vector with 50 nM miR-574-3p mimic or scrambled sequences with Lipofectamine 2000 reagent. Finally, the cells were harvested and then lysed with cell lysis buffer 48 h later. Luciferase activity of the protein was assayed on the Dual luciferase reporter assay instrument (Promega) by following the instructions provided. The luciferase activity of firefly was used as the control assay.

### Cell viability assay

The cell proliferative ability undergone various treatments was measured with Cell Counting Kit-8 (CCK-8) (Dojindo, Japan). The cells (1 × 10^4^) treated with miR-574-3p mimics or CCND2-siRNA were seeded in 96-well plates respectively and individually incubated for 24, 48 or 72 h, respectively. After incubation for 72 h, CCK-8 solution was pipetted into each well and treated for 60 min in a cell incubator at 37°C. Then, the absorbance at 450 nm per hole was recorded by ELIASA (Rayto Life and Analytical Science C. Ltd., Shenzhen, China).

### Edu Detection

SW480 and HT29 cells were split and seeded into 96-well plates and treated with miR-574-3p mimics or CCND2-siRNA. Forty-eight hours later, EdU 100 μm (Cell Light EdU DNA imaging Kit; Guangzhou RiboBio, China) was pipetted to each well, which were then lasted for 2 h. The cells were stained as mentioned previously. Apollo®643 enzymes Azide staining and flow cytometry were applied for analysis, and for identification of Edu positive cells as well.

### Apoptosis detection

Cells (1 × 10^7^) were centrifuged, separated and washed with cold PBS, which were followed by staining with Annexin V-FITC + 1 mg/ml PI, and cells were analyzed by FACS Calibur flow cytometry (Becton-Dickinson, Franklin Lakes, NJ, U.S.A.). Annexin V-FITC(+)/PI(+) and Annexin V-FITC(+)/PI(-) staining were used to identify cell apoptosis at early or late stage, respectively.

Apoptotic cells were detected with Hoechst 33342 nuclear staining. Cells were seeded on 6-well plates and maintained with Hoechst 33342 blue fluorescent nuclear dye (Sigma) for 30 min, fluorescence microscopy was applied to detect nuclear morphology of the cells and Hoechst 33342 staining was detected at 365 nm.

### Transwell assay

The migration assay of 1 × 10^4^ cells was carried out in an uncoated Transwell chamber without serum medium. Similarly, the invasion assay was carried out with cells suspension in serum-free medium in a Transwell chamber, the upper chamber of which was covered with artificial basement membrane. Cotton swabs were applied to take out of the non-migrated or non-invasive cells, which have been stained with Crystal Violet and then they were counted under inverted microscope.

### Electrophoretic mobility shift assay (EMSA)

EMSAs were conducted with the advanced DIG Gel Shit kit (Roche Diagnostics, Mannheim, Germany) according to instructions. The containing CCND2-binding sites double-strand oligonucleotide probes were produced by Shanghai Sangon (Shanghai, China). The nuclear fractions of SW480 and HT29 cell lysates were isolated with CelLytic™ nuclear™ Extraction kits (Sigma) in compliance with the manufacturer’s manual. The EMSA detection method is as mentioned before. Oligonucleotides were electroblotted onto nylon membranes with positive charge (Roche Diagnostics, Indianapolis, IN, U.S.A.), followed by immunodetection with anti-digoxin-AP (Roche Diagnostics).

### Statistical analysis

The data collected were statistically evaluated and analyzed with SPSS Ver.18.0 (Chicago, IL, U.S.A.). All the data are expressed as mean ± SD. The statistical significance of the variances of different groups was determined after ANOVA or paired/unpaired Student’s *t*-test. *P* value < 0.05 was considered as statistically significant difference.

## Results

### MiR-574-3p expressions in CRC tissues and cell lines

qRT-PCR results revealed the relatively lower expression level of miR-574-3p in 62 tumor tissues of patients than that in corresponding control tissues (Figure 1A). Also, the miR-574-3p expression was down-regulated in CRC cell lines by comparison with NCM460 cells (Figure 1B). This potentiated miR-574-3p as an important regulator in human CRC, which laid a foundation for our further *in vitro* investigations.

**Figure 1:** Expression of miR-574-3p in CRC cell lines and tissues The relative levels of miR-574-3p expression in human CRC cell lines and tissues were assayed by qRT-PCR. (**A**) The relative expression of miR-574-3p in human CRC tissues and the corresponding control tissues without metastasis. (**B**) The relative level of miR-574-3p expression in human CRC cell lines; *P < 0.05, **P < 0.01, ***P <0.001.

### Clinicopathological characteristics and miR-574-3p expression levels of CRC patients

Table 1 summarized the clinicopathological parameters of 62 patients with CRC recruited in this investigation in details. Patients were assigned into two different groups according to their median expression value of miR-574-3p. It was illustrated that miR-574-3p expression level was correlated with the tumor size (*P* = 0.008) and advanced clinical stage (*P* < 0.001), and distant metastasis (*P* = 0.0148). However, no correlation was found between the miR-574-3p expression level and age, gender or tumor location (*P* > 0.05).

### MiR-574-3p overexpression inhibited proliferation of CRC cells

It was found that miR-574-3p was overexpressed after miR-574-3p mimics was transfected into SW480 and HT29 CRC cells (*P* < 0.001; Figure 2A). The proliferation of SW480 and HT29 cells treated with miR-574-3p mimics was inhibited by comparison with NC group cells (Figure 2B). In contrast, treatment with miR-574-3p inhibitor significantly increased the viability of SW480 and HT29 cells (Figure 2C,D). Furthermore, EdU results indicated that the proliferative rate of SW480 and HT29 cells that overexpressed miR-574-3p decreased significantly (Figure 2E).

**Figure 2:** miR-574-3p is a blocker of CRC cell proliferation (**A**) miR-574-3p was overexpressed in SW480 and HT29 cells. (**B**) The proliferative rates of SW480 and HT29 cells transfected with miR-574-3p mimics detected by CCK-8 assay. (**C**) The expression of miR-574-3p in SW480 and HT29 cells treated with miR-574-3p inhibitor. (**D**) The proliferative rates of SW480 and HT29 cells transfected with miR-574-3p inhibitor detected by CCK-8 assay. (**E**) Cell proliferative rates determined by EdU flow cytometry assay; *P < 0.05, **P < 0.01, ***P < 0.001.

### MiR-574-3p overexpression inhibited cell migration and invasion of CRC cells

The effects of miR-574-3p expression on migration or invasiveness ability of CRC cells were detected by Transwell assay. Our data showed that the migrative and invasive rates of SW480 and HT29 cells treated with miR-574-3p mimics were dramatically inhibited by comparison with those treated with scrambled sequences (Figure 3A,B). On the contrary, transfetion with miR-574-3p inhibitor remarkably suppressed the migration and invasion of SW480 and HT29 cells (Figure 3C,D).

**Figure 3:** miR-574-3p is a suppressor of CRC cell migration and invasion (**A** and **B**) Effects of miR-574-3p mimics on the migration and invasion of SW480 and HT29 cells were detected by Transwell assay (×40 magnification). (**C** and **D**) Effects of miR-574-3p inhibitor on the migration and invasion of SW480 and HT29 cells were detected by Transwell assay; **P < 0.01.

### MiR-574-3p overexpression induced apoptosis of CRC cells

The present study applied Annexin V-FITC/PI staining method to explore the influence of miR-574-3p on the cell apoptosis of SW480 and HT29 cells. The acquired results demonstrated that miR-574-3p mimics significantly increased the apoptotic rate of SW480 and HT29 cells (Figure 4A,B). Further, Hoechst 33342 nuclear staining showed that SW480 and HT29 cells transfected with miR-574-3p mimics had higher apoptotic rate than those transfected with scrambled sequences (Figure 4C).

**Figure 4:** Overexpressed miR-574-3p promoted apoptosis in CRC cells (**A** and** B**) CRC cell apoptosis was detected by flow cytometry analyses after miR-574-3p mimics transfection. (**C**) The percentages apoptotic rates in each experimental group were qualified Hoechst staining; *P < 0.05, **P < 0.01.

### CCND2 was the direct target of miR-574-3p

Western blotting results found that CCND2 protein expression levels were up-regulated in both CRC specimen and CRC cell lines compared with the corresponding controls (Figure 5A). Furthermore, the expressive levels of CCND2 mRNA in SW480 and HT29 cells treated with miR-574-3p mimics or inhibitor were assayed with qRT-PCR. The results denoted the relatively lower expression of CCND2 mRNA in SW480 and HT29 cells than the cells transfected with miR-574-3p mimics (Figure 5B), whereas treatment with miR-574-3p inhibitor showed opposite results (Figure 5C). Western blot results showed that the miR-574-3p overexpression inhibited the expression of CCND2 protein (Figure 5D). In summary, these results suggested that the mRNA and protein expression levels of CCND2 were both inhibited by miR-574-3p.

**Figure 5:** CCND2 is a direct target of miR-574-3p (**A** and **B**) CCND2 protein expression in human CRC tissues (T) and control tissue (**C**) or human CRC cell lines were detected by Western blot analysis. (**B**) The relative expression levels of CCND2 mRNA in SW480 and HT29 cells treated with miR-574-3p mimics were measured by qRT-PCR. (**C**) The mRNA levels of CCND2 in SW480 and HT29 cells treated with miR-574-3p inhibitor were determined by qRT-PCR. (**D**) CCND2 protein expression decreased in SW480 and HT29 cells by treatment with miR-574-3p mimics. (**F**) Luciferase activity was significantly decreased in CCND2-WT group compared with CCND2-Mut group after treatment with miR-574-3p mimics. (**G**) CCND2 expression in SW480 cells transfected with miR-574-3p mimics alone or together with CCND2. (**H**) Cell viability of SW480 cells transfected with miR-574-3p mimics alone or together with CCND2. (**I**) The migration and invasion activities of SW480 cells transfected with miR-574-3p mimics alone or together with CCND2; *P < 0.05, **P < 0.01.

In order to determine whether CCND2 is a target gene of miR-574-3p, we applied Target Scan (http://www.targetscan.org/vert_72/) and miRDB (www.mirdb.org) to conduct bioinformatics analysis, and it demonstrated that miR-574-3p possessed a predictive potential in human CCND2 3′-UTR (Figure 5E). Then, the luciferase reporter system detection was performed and CCND2 was tested as the direct docking gene of miR-574-3p. The findings illustrated that the luciferase activity of the reporter was inhibited by miR-574-3p mimics. However, the luciferase activity between the CCND2 Mut group and the control group showed no statistical changes (*P* > 0.05, Figure 5F). All of the investigations demonstrated that the miR-574-3p blocked the expression of CCND2 through directly regulating the 3′-UTR region of CCND2. Next, we investigated whether CCND2 plays a role in the action of miR-574-3p. We found that overexpression of CCND2 blocked the inhibitory effects of miR-574-3p mimics on the growth, migration and invasion of SW480 cells (Figure 5G–I). These results indicated that miR-574-3p suppressed CRC progressing by down-regulation of CCND2.

## Discussion

Accumulative studies suggest that microRNAs have been implicated in regulating angiogenic responses in normal and cancer cells [9,10]. Moreover, recent investigations support the role of microRNAs in the occurrence and development of human cancers [11]. Thus, the dysregulation of microRNAs would contribute to the progression of cancer [12]. Since that miRNAs exert their functions through regulating targeted mRNAs, therefore, it is essential to understand their function by identification of miRNA targets.

Our study indicated that up-regulation of miR-574-3p had prohibited the cell proliferation of human CRC cells *in vitro* and increased the apoptosis level via targeting CCND2. We uncovered the reduction of miR-574-3p expression in CRC tissue samples and cell lines. Additionally, the overexpression of miR-574-3p blocked the cell proliferation and migration of CRC cells, as well as promoted cell apoptosis. The treatment of mir-574-3p mimics on CRC cells reduced the expression of CCND2 protein, suggesting that CCND2 is the target gene of mir-574-3p. Additionally, the down-regulation of CCND2 inhibits the proliferation and migration of CRC cells, which promote cell apoptosis.

Abnormal expression of miRNA has been found in various human cancer types. The genes encoding miR-574-3p are located on chromosomes 4P (4p14 and 4p15) with a tumor inhibitory miRNA function [13]. MiR-574-3p expression levels were decreased in spinal chordoma patients [14]. Overexpression of miR-574-3p prohibited the cell proliferation of osteosarcoma cancer cells, promoting cell death via targeting by targeting SMAD4 signaling pathway [15]. It has been reported that miR-574-3p blocked the epithelial–mesenchymal transition (EMT) and promoted cisplatin sensitivity through inhibiting the activity of zinc finger E-box binding homeobox transcription factor 1 (ZEB1) in GC cells [16].

The present study potentiated the role of miR-574-3p in blocking the cell proliferation of human CRC cells *in vitro* through targeting CCND2, which increases cell apoptosis. CCND2 is a type of cell cycle regulatory gene of great value, the abnormal expression of which could result in abnormal cell proliferation. Previously, CCND2 was demonstrated as an abnormally expressed in pancreatic cancer, colorectal cancer and prostate cancer [17–19]. The present study proved the significant increase in the expression of CCND2 gene and protein in CRC tissues and cell lines. In addition, CCND2 expression was knocked down with RNA interference, which prohibited the cell proliferation and migration of CRC cells and related to the increase of cell apoptosis level. Taken together, our study demonstrated that the down-regulation of miR-574-3p through CCND2-mediated signaling pathway promotes the proliferation of human CRC cells.

## Conclusion

In conclusion, the present study suggests that the up-regulation of miR-574-3p may increase the apoptotic level of human CRC cells via targeting CCND2 to inhibit the proliferation of human CRC cells. Our study demonstrated that miR-574-3p was a potential therapeutic and prognostic biomarker in human CRC.

## Abbreviations

CCND2: Cyclin D2
CRC: colorectal cancer
EMSA: electrophoretic mobility shift assay
EMT: epithelial–mesenchymal transition
ZEB1: zinc finger E-box binding homeobox transcription factor 1

## References

[1] JemalA., BrayF., CenterM.M., FerlayJ., WardE. and FormanD. (2011) Global cancer statistics. CA Cancer J. Clin. 61, 69–90 10.3322/caac.2010721296855

[2] SiegelR.L., MillerK.D. and JemalA. (2015) Cancer statistics, 2015. CA Cancer J. Clin. 65, 5–29 10.3322/caac.2125425559415

[3] BartelD.P. (2004) MicroRNAs: genomics, biogenesis, mechanism, and function. Cell 116, 281–297 10.1016/S0092-8674(04)00045-514744438

[4] WangS., WangL., BayaxiN., LiJ., VerhaeghW., JanevskiA.et al. (2013) A microRNA panel to discriminate carcinomas from high-grade intraepithelial neoplasms in colonoscopy biopsy tissue. Gut 62, 280–289 10.1136/gutjnl-2011-30155422535378

[5] LodishH.F., ZhouB., LiuG. and ChenC.Z. (2008) Micromanagement of the immune system by microRNAs. Nat. Rev. Immunol. 8, 120–130 10.1038/nri225218204468

[6] OkugawaY., ToiyamaY. and GoelA. (2014) An update on microRNAs as colorectal cancer biomarkers: where are we and what’s next? Expert Rev. Mol. Diagn. 14, 999–1021 10.1586/14737159.2014.94690725163355PMC4374444

[7] HongL., HanY., YangJ., ZhangH., ZhaoQ., WuK.et al. (2014) MicroRNAs in gastrointestinal cancer: prognostic significance and potential role in chemoresistance. Expert Opin. Biol. Ther. 14, 1103–1111 10.1517/14712598.2014.90778724707835

[8] SchetterA.J., LeungS.Y., SohnJ.J., ZanettiK.A., BowmanE.D., YanaiharaN.et al. (2008) MicroRNA expression profiles associated with prognosis and therapeutic outcome in colon adenocarcinoma. JAMA 299, 425–436 10.1001/jama.299.4.42518230780PMC2614237

[9] CaiY., YuX., HuS. and YuJ. (2009) A brief review on the mechanisms of miRNA regulation. Genomics Proteomics Bioinformatics 7, 147–154 10.1016/S1672-0229(08)60044-320172487PMC5054406

[10] WangY.Q., RenY.F., SongY.J., XueY.F., ZhangX.J., CaoS.T.et al. (2014) MicroRNA-581 promotes hepatitis B virus surface antigen expression by targeting Dicer and EDEM1. Carcinogenesis 35, 2127–2133 10.1093/carcin/bgu12824913918

[11] LiuQ., XuY., WeiS., GaoW., ChenL., ZhouT.et al. (2015) miRNA-148b suppresses hepatic cancer stem cell by targeting neuropilin-1. Biosci. Rep. 35, 42 10.1042/BSR20150084PMC461367225997710

[12] AnticaM., KusicB., HranilovicD., DietzA.B. and Vuk-PavlovicS. (2002) Cloning the cDNA for murine U2 snRNP-A’ gene and its differential expression in lymphocyte development. Immunol. Lett. 82, 217–223 10.1016/S0165-2478(02)00064-012036604

[13] YangH., ZhangJ., LiJ., ZhaoF., ShenY. and XingX. (2018) Overexpression of miR-574-3p suppresses proliferation and induces apoptosis of chronic myeloid leukemia cells via targeting IL6/JAK/STAT3 pathway. Exp. Therap. Med. 16, 4296–43023034470310.3892/etm.2018.6700PMC6176133

[14] ZouM.X., GuoK.M., LvG.H., HuangW., LiJ., WangX.B.et al. (2018) Clinicopathologic implications of CD8(+)/Foxp3(+) ratio and miR-574-3p/PD-L1 axis in spinal chordoma patients. Cancer Immunol. Immunother. 67, 209–224 10.1007/s00262-017-2080-129051990PMC11028121

[15] XuH., LiuX., ZhouJ., ChenX. and ZhaoJ. (2016) miR-574-3p acts as a tumor promoter in osteosarcoma by targeting SMAD4 signaling pathway. Oncol. Lett. 12, 5247–5253 10.3892/ol.2016.535528105233PMC5228465

[16] WangM., ZhangR., ZhangS., XuR. and YangQ. (2019) MicroRNA-574-3p regulates epithelial mesenchymal transition and cisplatin resistance via targeting ZEB1 in human gastric carcinoma cells. Gene 700, 110–119 10.1016/j.gene.2019.03.04330917930

[17] XuM., ChenX., LinK., ZengK., LiuX., PanB.et al. (2018) The long noncoding RNA SNHG1 regulates colorectal cancer cell growth through interactions with EZH2 and miR-154-5p. Mol. Cancer 17, 141 10.1186/s12943-018-0894-x30266084PMC6162892

[18] ChenY., ZhangQ., WangQ., LiJ., SipekyC., XiaJ.et al. (2017) Genetic association analysis of the RTK/ERK pathway with aggressive prostate cancer highlights the potential role of CCND2 in disease progression. Sci. Rep. 7, 4538 10.1038/s41598-017-04731-428674394PMC5495790

[19] HuW., LiuQ., PanJ. and SuiZ. (2018) MiR-373-3p enhances the chemosensitivity of gemcitabine through cell cycle pathway by targeting CCND2 in pancreatic carcinoma cells. Biomed. Pharmacother. 105, 887–898 10.1016/j.biopha.2018.05.09130021382

